# The Chemokine CXCL13 Is a Prognostic Marker in Clinically Isolated Syndrome (CIS)

**DOI:** 10.1371/journal.pone.0011986

**Published:** 2010-08-05

**Authors:** Johannes Brettschneider, Anne Czerwoniak, Makbule Senel, Lubin Fang, Jan Kassubek, Elmar Pinkhardt, Florian Lauda, Tamara Kapfer, Sarah Jesse, Vera Lehmensiek, Albert C. Ludolph, Markus Otto, Hayrettin Tumani

**Affiliations:** Department of Neurology, University of Ulm, Ulm, Germany; Julius-Maximilians-Universität Würzburg, Germany

## Abstract

**Background:**

There is increasing recognition of the importance of B lymphocytes in the immunopathogenesis of multiple sclerosis (MS), encouraging the evaluation of B cell-associated biomarkers in the cerebrospinal fluid (CSF). We aimed to evaluate the relevance of the B cell chemoattractant CXCL13 as a prognostic marker in patients with clinically isolated syndrome (CIS) regarding conversion to MS, and to compare it to Barkhof criteria in magnetic resonance imaging (MRI), oligoclonal bands (OCB) and the polyspecific intrathecal B cell response against measles, rubella and varicella zoster virus (MRZR).

**Methodology/Principal Findings:**

CXCL13 was determined in a prospective study over 2 years including 46 patients that remained CIS over follow-up (CIS-CIS), 45 patients that developed MS (CIS-RRMS), and 30 controls using ELISA. CSF CXCL13 was significantly elevated in CIS-RRMS as compared to CIS-CIS and controls (p<0.001). It was significantly elevated in CIS with OCB (p<0.001), positive MRZR (p = 0.04), and gadolinium enhancement in MRI (p = 0.02) and showed a significant correlation with CSF leukocyte count (p<0.001) and QIgG (p<0.001). CXCL13 showed the best positive predictive value (PPV) of all parameters investigated (70%, 95%-CI: 53–84%), which could be further increased by combination with Barkhof criteria in MRI (80%).

**Conclusions/Significance:**

Our data indicate the relevance of CXCL13 in CIS to predict conversion to MS. It furthermore shows CXCL13 to be an important mediator in the inflammatory cascade associated with the polyspecific intrathecal B cell response that manifests itself in OCB and MRZR.

## Introduction

In most patients who develop multiple sclerosis (MS), the disease initially manifests itself in a first relapse-like episode known as clinically isolated syndrome (CIS) [1]. Given the importance of an early treatment of MS, the challenge in patients with CIS is to identify those at high risk of future events that would confirm the diagnosis of MS [2], [3]. Consequently, there is an ongoing search for biomarkers that could help to evaluate the prognosis in CIS [1], [4], [5], [6]. Increasing recognition of the importance of B lymphocytes in the pathogenesis of MS [7] encouraged the evaluation of B cell-associated biomarkers in the cerebrospinal fluid (CSF) of patients with MS and CIS. CSF oligoclonal bands (OCB) were shown to be an independent risk factor in CIS implementing an almost two-fold increased risk of having a second relapse [8]. Furthermore, we could demonstrate the polyspecific intrathecal B cell response against the neurotropic viruses measles, rubella and varicella zoster (“MRZ reaction”, MRZR) to be of prognostic relevance in CIS [9]. A key regulator of B cell recruitment in MS is the chemokine CXCL13 [7]. It belongs to the CXC chemokine family and is a selective chemoattractant for B lymphocytes and B helper T cells via its specific receptor CXCR5 [10]. CXCL13 was found to be present in active MS lesions and to be elevated in CSF of MS and CIS [11], [12], [13]. However, previous studies included only small numbers of patients with CIS (n = 22 [11], n = 25 [13]) and provided no longitudinal clinical data on the prognostic relevance of CSF CXCL13 regarding conversion to MS. We aimed to evaluate the relevance of CXCL13 as a prognostic marker in CIS and to compare it to established parameters like Barkhof criteria in magnetic resonance imaging (MRI) [14], OCB and MRZR.

## Methods

### Patients

In a prospective study of the Department of Neurology, University of Ulm (Germany), we collected paired CSF and serum samples from patients with CIS that remained CIS (CIS-CIS) over a follow-up of 2 years and from patients with CIS that developed definite MS of the relapsing-remitting subtype (CIS-RRMS) over the same period [2] (Table 1). Disability was rated using Kurtzke's Expanded Disability Status Scale (EDSS) [15] by two experienced neurologists in our department (HT and FL), each unaware of any results on the CSF biomarkers. Lumbar puncture was performed as part of the routine diagnostic work up using a atraumatic 22G Sprotte needle and prior to application of steroids in all patients. The control group consisted of 30 age-matched patients who presented with infrequent episodic tension-type headache [16] and showed no evidence of a structural, haemorrhagic or inflammatory lesion in MRI.

**Table 1:** Demographic data, CSF, serum and MRI findings in patients with clinically isolated syndrome (CIS) and controls.

	CIS all	CIS-CIS	CIS-RRMS	CTRL	S*
**n (female/male)**	91 (53/38)	46 (27/19)	45 (24/21)	30 (19/11)	NS
**Age [years]**	34 (13–77)	37 (17–77)	33 (13–55)	36 (15–71)	NS
**EDSS**	2 (0–6)	2 (0–6)	2.5 (0–5)	-	NS
**CSF cells/**µ**L**	5 (0–86)	4 (0–86)	7 (0–29)	1 (0–4)	NS
**Qalb**	5.2 (1.5–14.7)	5.0 (2.4–11.8)	5.4 (1.5–14.7)	4.1 (2.3–8.5)	NS
**QIgG**	3.4 (1.5–14.8)	2.9 (1.5–10.8)	3.9 (1.8–14.8)	2.0 (0.9–4.2)	NS
**CSF CXCL13 [pg/ml]**	3.7 (0–64.4)	1.6 (0–56.1)	9.3 (0–64.4)	0 (0–5.1)	p = 0.008
**Serum CXCL13 [pg/ml]**	30.7 (8.6–528.8)	36.1 (12–528.8)	30 (8.6–84.8)	33.3 (13.4–357.5)	NS
**MRZR**	34	26	42	0	p = 0.04
**OCB**	78	63	91	0	p = 0.003
**Barkhof criteria**	15	5	25	0	p = 0.002

Barkhof criteria = 3 of 4 criteria fulfilled, CIS all = all patients with CIS, CIS-CIS = patients with CIS that remained CIS over follow-up, CIS-RRMS = CIS patients with conversion to MS over follow-up, CTRL = controls, EDSS = Kurtzke Expanded Disability Status Scale, MRZR = antibody indexes (AI) for measles, rubella, zoster, two or more AI≥1.5, OCB = oligoclonal bands in cerebrospinal fluid only, Qalb = albumin CSF/serum concentration ratio, QIgG = IgG CSF/serum concentration ratio, NS = not significant, S = statistical significance, * CIS-CIS vs. CIS-RRMS.

Relative frequencies (%) are given for discrete variables, median and range for continuous variables.

### Ethics statement

Written informed consent was obtained from all patients in accordance with the Declaration of Helsinki, and the study was approved by the ethics committee of the University of Ulm.

### CSF basic analysis and determination of MRZR

Samples were handled in accordance with the BioMS guidelines [17]. CSF leukocyte count (cells/cu.mm), total protein (g/L), lactate (mmol/L), the albumin CSF/serum concentration ratio (Q_alb_), immunoglobulins G, A and M, and OCB were obtained as previously described [18], [19], [20]. Antibody levels against measles, rubella and zoster were determined using an enzyme-linked immunosorbent assay (ELISA) according to the instructions as supplied by the manufacturer (Genzyme Virotech, Rüsselsheim, Germany) [9]. Quantitative expression of the intrathecal immune response was based on calculation of the CSF/serum quotients (Q) of specific antiviral IgG antibodies (IgG[spec]) and total IgG (IgGtotal): QIgG[spec] = IgGspec[CSF]/IgGspec[serum], and QIgG[total] = IgGtotal[CSF]/IgGtotal[serum]). The intrathecal synthesis of antibodies was detected by calculation of the corresponding antibody indices (AI): AI = QIgG[spec]/QIgG[total] (Figure 1). In case of an overall intrathecal Ig synthesis above the reference range (Qlim), Qlim was used instead of QIgG[total]: AI = QIgG[spec]/Qlim, if QIgG[total]>Qlim [21]. The upper reference range of QIgG[total], Qlim, was calculated according to Reiber's formula [21]. AI values ≥1.5 were considered to be indicative of intrathecal IgG synthesis against the respective antigen [21], [22], [23]. MRZR was considered positive if two or more AI values were ≥1.5.

**Figure 1:** Reiber diagram and antibody index. Left side: Reiber diagram visualizing intrathecal IgG synthesis using a double-logarithmic scaling to present the IgG CSF to serum quotient (QIgG) in relation to the albumin CSF to serum quotient (Qalb), and showing the hyperbolic function Qlim that indicates the upper reference range of QIgG. In the upper right corner of the diagram, the relative extent of intrathecal IgG synthesis is indicated. Right side: Formula for antibody index (AI) and Qlim.

### Determination of CXCL13

CXCL13 was measured using ELISA (Quantikine; R&D Systems, Minneapolis, MN) according to the instructions as supplied by the manufacturer. Samples of 50 µl CSF and 50 µl serum were used for the ELISA. Details on the application of the assay for CSF have been published previously by our group [24].

### MRI analysis

MRI scans of the brain and spinal cord were performed on a 1.5 tesla whole-body MRI (Symphony Siemens, Erlangen, Germany) according to a previously fixed protocol including T1-weighted spin-echo (SE) axial slices with and without application of gadolinium-DTPA (Gd) as well as T2-weighted SE axial slices. Hyperintense lesions on T2-weighted MRI>3 mm^2^ were analyzed and quantified. Barkhof criteria [14] were considered to be positive if three of four criteria were fulfilled according to the standard procedure.

### Statistical analysis

Absolute and relative frequencies were given for discrete variables, median and range for continuous variables. Differences between CIS-CIS and CIS-RRMS were analyzed by Chi-Square test and Mann-Whitney U-Test respectively on a univariate basis in an exploratory sense. To compare raw data of multiple groups, a non-parametric ANOVA (Kruskal-Wallis analysis of variance on ranks) was applied, followed in case of significance by Dunn's Method. All correlations were studied using Spearman's rank correlation coefficient. P-values below 0.05 were considered to be significant. Sensitivity was calculated as (true-positive/[true-positive+false-negative]), specificity was calculated as (true-negative/[true-negative+false-positive]). The positive predictive value (PPV) was calculated as (true-positive/[true-positive+false-positive]), and the negative predictive value (NPV) as (true-negative/[true-negative+false-negative]). For all diagnostic values the exact 95% confidence intervals were given [25]. To examine the accuracy of CXCL13 to differentiate CIS-CIS and CIS-RRMS, we used Receiver Operating Characteristic (ROC) analysis, calculating the area under the ROC curve (AUROCC). The Youden index was calculated to determine the cut-off value which maximizes discriminating accuracy [26].

## Results

Of 91 patients with CIS, 45 developed MS over a follow-up of two years (conversion rate 49.5%). There was no significant difference regarding age, gender and EDSS distribution between patients with CIS-RRMS and CIS-CIS at onset of study (Table 1). MRZR was observed to be positive in 34% of all patients with CIS (Table 1). It was significantly more frequent in CIS-RRMS as compared to CIS-CIS (p = 0.04), as were positive OCB in CSF (p = 0.003) and Barkhof criteria in MRI (p = 0.002).

We observed a significant difference of CSF CXCL13 between patients with CIS-CIS, CIS-RRMS and controls (p<0.001, Kruskal-Wallis analysis of variance on ranks, Figure 2), with post-hoc analysis (Dunn's Method) showing CSF CXCL13 to be significantly elevated in CIS-RRMS as compared to CIS-CIS and controls and to be elevated in CIS-CIS as compared to controls (p<0.05 each). In contrast, no significant difference of serum CXCL13 concentrations was observed between the groups (p = 0.08).

**Figure 2:** CXCL13 in patients with CIS. A) Boxplot shows CSF concentrations of CXCL13 in patients with CIS-CIS (patients with CIS that remained CIS over follow-up of two years), CIS-RRMS (CIS patients with conversion to MS over follow-up) and controls (CTRL). P-value refers to comparison of CIS-CIS, CIS-RRMS and controls. B) Boxplot shows CSF concentrations of CXCL13 in CIS patients with and without oligoclonal bands (OCB) in CSF. P-value refers to comparison of CIS patients with and without OCB. C) Boxplot shows CSF concentrations of CXCL13 in CIS patients with and without positive MRZR (“MRZ reaction”, intrathecal antibody production against measles, rubella and varicella zoster, with two antibody indices ≥1.5). P-value refers to comparison of CIS patients with and without MRZR. D) Boxplot shows CSF concentrations of CXCL13 in CIS patients with and without gadolinium-enhancing lesions in T1-weighted MRI. P-value refers to comparison of CIS patients with and without gadolinium-enhancing lesions. A)–D) The box represents the 25^th^ to 75^th^ quartile, the whiskers represent the range, and the horizontal line in the box represents the median. Black dots beyond the whiskers indicate outliers, d = number of patients with detectable CXCL13 concentrations in CSF.

CSF CXCL13 was significantly higher in patients with presence of OCB in CSF as compared to patients who did not show OCB in CSF (p<0.001). Similarly, it was significantly higher in CIS with positive MRZR as compared to CIS without MRZR (p = 0.003, Figure 2).

CSF CXCL13 showed a significant correlation with CSF leukocyte count (p<0.001, R = 0.59, Figure 3) and with CSF plasma cells count (p = 0.03, R = 0.31). In addition, we observed a significant correlation of CSF CXCL13 with the extent of intrathecal IgG synthesis as measured by the CSF/serum ratio of IgG (QIgG, p<0.001, R = 0.57). In contrast, no correlation of CSF CXCL13 with blood-CSF barrier function as measured by Q_alb_ was detectable (p = 0.25). We also found no correlation of CSF CXCL13 with age of CIS patients (p = 0.56). Furthermore, no correlation with duration from onset of symptoms to lumbar puncture was observed (p = 0.13). We found CSF CXCL13 to be significantly elevated in patients who showed Gd-enhancing lesions in T1-weighted MRI (p = 0.02). ROC analysis followed by application of the Youden index revealed 7.7 pg/ml as optimal cut-off value to differentiate between CIS-CIS and CIS-RRMS (AUROCC 0.64).

**Figure 3:** Relation of CXCL13 to cell count. Dot plot shows CSF CXCL13 in patients with CIS plotted against CSF leucocyte count. Straight line represents regression line; correlation was significant (p<0.001, R = 0.59).

Of all markers investigated, OCB showed the highest sensitivity for conversion of CIS to MS (91%), which could not be improved by adding any of the other parameters (Table 2). Barkhof criteria (92%) [14] showed the highest specificity of all single parameters. CXCL13 showed the best PPV (70%) for predicting conversion from CIS to MS of all single parameters, and was superior to Barkhof criteria (67%) and MRZR (64%). PPV could be increased to 80% by combination of CXCL13 with Barkhof criteria in MRI (Table 2).

**Table 2:** Sensitivity, specificity, positive (PPV), and negative (NPV) predictive value in percent (exact 95% confidence interval in brackets) for CSF and MRI parameters regarding conversion of clinically isolated syndrome to definite multiple sclerosis.

	Sensitivity	Specificity	PPV	NPV
**OCB**	91 (97–98)	36 (23–52)	59 (46–70)	81 (58–95)
**MRZR**	42 (25–61)	74 (55–88)	64 (41–83)	55 (39–70)
**CXCL13**	62 (46–76)	76 (61–87)	70 (53–84)	69 (54–81)
**Barkhof criteria**	17 (7–34)	92 (79–98)	67 (30–93)	55 (43–68)
**OCB+CXCL13**	60 (43–74)	78 (64–89)	71 (54–85)	63 (54–80)
**OCB+MRZ**	39 (23–58)	74 (55–88)	62 (38–82)	53 (38–69)
**OCB+Barkhof**	17 (6–33)	95 (82–99)	75 (35–97)	55 (42–67)
**CXCL13+MRZ**	32 (17–51)	90 (74–98)	77 (46–95)	57 (42–71)
**CXCL13+Barkhof**	12 (3–27)	98 (87–100)	80 (28–99)	57 (44–68)
**MRZ+Barkhof**	7 (1–24)	96 (80–100)	67 (9–99)	49 (34–64)

Barkhof = 3 of 4 Barkhof criteria fulfilled, MRZR = antibody indexes (AI) for measles, rubella, zoster, two or more AI≥1.5, OCB = oligoclonal bands in cerebrospinal fluid only.

## Discussion

Our observation of elevated CSF CXCL13 in CIS is in line with previous studies that found CXCL13 to be elevated in CSF and serum across different subtypes of MS as well as in CIS [11], [12], [27], [28]. CXCL13 was shown to be present in active inflammatory lesions in MS [12]. It was suggested to derive from infiltrating macrophages, whereas in some patients with a secondary progressive course of disease (SPMS) it may also be produced by follicle-like structures in the leptomeninges [7], [12]. Leukocyte recruitment in MS is tightly regulated and involves sequential interactions between adhesion molecules, chemokines like CXCL13, and their specific receptors [29]. CXCR5 was shown to be present on B cells, as well as on a subset of T cells in blood and lymphatic tissue [30]. Consequently, CXCL13 is likely to play a key role in the regulation of B cell migration to the inflamed CNS [12], [29]. It furthermore was suggested to influence the cytokine environment in MS including an auto-regulatory loop via up-regulation of membrane LTa1b2 on B cells [31].

The correlation of CSF CXCL13 with leukocyte count, plasma cell count and QIgG confirms previous observations who found CSF CXCL13 to correlate with inflammatory disease activity in MS, especially intrathecal Ig production and accumulation of B and T cells in the CSF [12]. Our observation of elevated CSF CXCL13 in CIS patients with presence of OCB and positive MRZR (Figure 2) demonstrates the association of CXCL13 with the polyspecific intrathecal B cell response in MS, which was suggested to derive from long-lived plasma cells in an enhanced B cell-promoting environment [7]. While B cells produce pro-inflammatory cytokines such as IL-6, IL-12 and lymphotoxin, and play a role in antigen-presentation [32], they were also reported to have tissue-protective and anti-inflammatory capacities in MS including the release of neurotrophic factors such as nerve growth factor or brain-derived neurotrophic factor [33], [34]. Consequently, the elevation of B cell-associated markers like CXCL13 in the CSF of patients with CIS could indicate a pro-inflammatory, B cell promoting environment as well as an upregulation of compensatory protective mechanisms [7]. Molecules involved in B-cell trafficking and survival like CXCL13 could be promising targets for immune intervention. They could furthermore contribute to biomarker patterns that could help to identify patients that respond to B cell orientated therapies like plasmapheresis.

CXCL13 is no disease-specific marker of MS or CIS: Particularly high concentrations of CSF CXCL13 can be found in patients with neuroborreliosis, which is the neuroinflammatory disease with the highest proportion of B cells in the CSF [24], [35]. Furthermore, CSF CXCL13 was found to be elevated in other inflammatory CNS diseases including viral meningitis and encephalitis [12], confirming its role as a suitable marker of B cell recruitment. Recent evidence also indicates that, apart from inflammatory CNS diseases, CSF CXCL13 may be of diagnostic and prognostic relevance in B cell lymphoma of the CNS [36].

Several candidate markers have been investigated as possible predictors of progression from CIS to MS [4], [6], [8], [14], [37], [38], [39], [40]. Besides history and clinical findings, magnetic resonance imaging (MRI) has become the preferred tool to evaluate the prognosis in CIS. However, as shown in a meta-analysis evaluating the use of MRI in MS, MRI studies tend to produce higher estimates of sensitivity and lower estimates of specificity particularly in short-term studies [41]. Cerebrospinal fluid (CSF) is a promising source of biochemical markers in CIS, since the CSF compartment is in close anatomical contact with the brain interstitial fluid, and reflects biochemical changes associated with the disease [42], [43]. The most relevant statistical parameters to predict conversion from CIS to MS are the predictive values (PPV, NPV): The patient's disease status (CIS-CIS or CIS-RRMS) is unknown and the clinician needs to determine whether a positive/negative test result (e.g. the presence or absence of Barkhof criteria in MRI) indicates that the patient really has/does not have MS. Our data showed CXCL13 to have the best PPV of all single parameters investigated and to be superior to Barkhof criteria [14], MRZR and OCB. In a previous study, we could demonstrate MRZR to be of prognostic relevance in CIS [9]. However, an important drawback of MRZR is that its determination currently requires the application of three different ELISA assays with at least 300 µL CSF and the same amount of serum necessary. A workable combined assay (e.g. a multiplex assay) to determine these antibodies is still not available. Consequently, the determination of CXCL13 is more practicable, as it requires a smaller amount of CSF and serum for a single assay. Furthermore, our data demonstrates CXCL13 to be superior to MRZR to identify CIS patients at high risk of conversion to MS.

In conclusion, this study underlines the prognostic relevance of CXCL13 to predict conversion to MS in patients with CIS. We observed a considerable overlap regarding CSF CXCL13 concentrations between the groups as well as a considerable overlap in confidence intervals for the predictive values. Furthermore, due to limitations regarding the number of patients included (n = 91), we observed large confidence intervals especially for the combined analysis of the different markers. Consequently, this study should be considered a pilot study that warrants further validation of CSF CXCL13 as a prognostic marker in a multi-center approach on a large cohort of patients with CIS. Even though, our data suggest that CIS patients that show high CXCL13 concentrations in CSF and fulfill Barkhof criteria in MRI are at high risk to develop MS and should therefore be candidates for an early treatment with an immunomodulatory therapy.
